This article has been retracted.

# Evaluation Method of Mixed Teaching Efficiency of College Teachers Based on Kirkpatrick Model

**DOI:** 10.1155/2022/8609387

**Published:** 2022-08-21

**Authors:** Fenglan Liang, Weiwei Shen, Hongwei Shi, Buqin Zheng

**Affiliations:** School of Information Engineering, Suqian University, Suqian 223800, China

## Abstract

Online teaching has become more prevalent in recent years as a result of the process of digitization and adaptation to the times. Classroom instruction is no longer just conducted in person offline. Online education has received a lot of promotion, especially in the wake of the epidemic's effects, and has evolved into a blended teaching model that combines the two modes. The old system of measuring the effectiveness of teaching is no longer reliable or scientific in assessing the new blended teaching model, and it has many flaws. A perfect system for evaluating the effects of blended learning must therefore be built. In order to more accurately assess the teaching impact of the blended teaching model, this study aims to build a more comprehensive system for evaluating blended teaching effects. This paper introduces the Kirkpatrick four-level evaluation model, which plays a significant role in the evaluation field, in order to achieve this goal. The experiments in this study compared the Kirkpatrick model with the AHP, which is frequently used in the evaluation. Online, offline, and blended teaching models were the subject of an experimental investigation. The experimental results demonstrated that each index combination's weights in the Kirkpatrick model and the AHP model of the blended teaching effect evaluation system were fairly close to one another. The evaluation indicators all center on the assessment of practical ability after class, which is consistent with their focus. The innovation evaluation of course papers has the highest weight, and the weight of evaluation indicators is greater than 0.15; the Kirkpatrick model has the lowest weight of the number of platform logins, with a weight value of 0.011, and the evaluation index of the teaching effect evaluation system based on AHP.

## 1. Introduction

Higher education has always played a significant role in China, but recent years have seen a focus on improving the standard of higher education. Online learning has gradually gained popularity and improved teaching outcomes. The online learning mode has advanced and developed significantly in recent years, particularly in light of the epidemic's effects. The “hybrid” teaching method, which combines online and offline modes, has continued to be promoted by many schools. A useful tool for managing instruction and keeping tabs on instruction quality, the evaluation of the teaching impact of college instructors provides insight into the impact of instructors in the classroom. However, the majority of conventional techniques for measuring the effectiveness of instruction, including AHP, the Delphi method, and developmental student evaluation, are only effective when used in offline classroom settings. The evaluation results for the impact of blended learning obtained using this method are not rational or scientific, and it has flaws such as unclear evaluation standards, an incomplete assessment of the learning effect, and an inaccurate assessment of online classrooms. It is therefore urgent to set up a fair evaluation system for the effect of blended teaching at this time in light of how to accurately, efficiently, scientifically, and reasonably evaluate the effect of blended teaching in colleges and universities.

There are many teaching effect evaluation systems now, which are constantly being revised and improved, and many scholars have made a series of related researches. Dharmawardene and Wijewardene research explored whether the speech performance was affected by different speech modes. The experiment results showed that the blended teaching mode has a better teaching effect. And there are some associations between learning modes and skills that can be used in the future course development for [1]. In order to study the factors that affect students' perception of teaching effectiveness and the influence of teachers' course attributes on teaching effect, Pandhiani used factor analysis to analyze students' evaluation of teachers in a school. And the experiment showed there is indeed a relationship that is very helpful for the evaluation of teaching effectiveness [2]. In order to study the impact of the hospital teaching plan and improve the teaching skills of residents, Nejad et al. evaluated residents from two aspects based on the Kirkpatrick model. The test results showed that residents have improved their attitude toward the teaching ability of resident doctors after participating in the workshop, and the experiment showed a good effect on the second evaluation level of the model [3]. In order to understand and evaluate the current actual situation, Villanueva et al. described the knowledge of teaching assessment practice in engineering programs across the country, exploring three related research questions. The experimental results showed that students' evaluation of teaching at the end of class (SET) is the most commonly used method [4]. The research of many scholars has made the evaluation results of teaching effect more and more scientific and effective. However, with the rise of blended teaching methods, the previous teaching effect evaluation schemes are not accurate and effective for the evaluation of blended teaching. In the online teaching mode, it is challenging for teachers to pay attention to students' learning circumstances, and both student and teacher enthusiasm are significantly lower than in the offline mode. The assessments produced by the evaluation of the blended teaching mode's educational impact will be unreliable if the traditional evaluation system is still used. As a result, this study introduced the offset model and investigated the blended teaching method's teaching evaluation system in more detail.

The Korotkoff evaluation model is currently the most widely used model in the world and plays an important role in the evaluation field. Many scholars have carried out a series of studies based on this model. In order to explore the use of the Kirkpatrick model to assess aircrew food safety training, a survey interview was conducted with the relevant personnel using the snowball technique by Abdelhakim et al. Research studies have shown that safety training was ineffective in certain areas, including learning outcomes and behavioral changes, which directly impacted the implementation of food safety practices [5]. Du took the recent 3-year project of a university teacher training center as the research topic. Through the analysis of the current common training effectiveness evaluation models, he discussed the institutional problems in the evaluation of teacher training effectiveness in Zhejiang colleges and universities. The experiments have proved the feasibility of the applying the Korotkoff Model to the university teacher training system [6]. In view of the deficiencies in the use of the offset model by evaluators, Cahapay conducted a descriptive analysis of the limitations of the offset model in higher education, and found three limiting themes: it tends to use lower-level models, rigid ignoring other important aspects of the assessment, and lack of evidence on causal chains between tiers [7]. Qualitative and quantitative evaluation of academic programs is essential to increase effectiveness and quality improvement, so Chellaiyan and Suliankatchi evaluated the learning outcomes and effects of research methods workshops for medical students. He used Korotkoff models to analyze experimental findings and concluded: Evaluations from the methods workshop provided insights into the results and modifications needed for future improvements [8]. Many scholars in the evaluation field often use the Kirkpatrick four-level model for evaluation experiments, and it is widely used in the evaluation field. Therefore, the Kirkpatrick model is a very good choice for the blended teaching evaluation system in this study.

This study introduced the Kirkpatrick model and built the evaluation system based on it when building the blended teaching effect evaluation system. As the survey object for the experimental investigation, a university was chosen. Fifteen well-known experts with professional standing were consulted in the experiment to examine the weights of the indicators in the developed evaluation system, and another common evaluation method was used to compare with the Kirkpatrick model put forth in this study. The experimental findings revealed a very close weight trend between the Kirkpatrick four-level evaluation model-based evaluation system and the AHP. The minimum index was the number of logins to the platform, the weight values were 0.011 and 0.022, and the innovation evaluation indicators were all greater than 0.15. It demonstrated the validity and precision of the Kirkpatrick model-based blended teaching effect evaluation system. Compared to the analytic hierarchy process, which has good research value, the steps for building the system were clearer and simpler.

## 2. Blended Teaching Effect Evaluation System

### 2.1. Evaluation Methods of Blended Learning

Online classroom teaching effect evaluation and offline classroom teaching effect evaluation must be used in a reasonable combination to assess the effectiveness of blended learning. Online and offline monitoring and evaluation are both conducted concurrently, and the process and result evaluation are combined [9]. It's important to examine blended learning from a variety of angles when assessing its impact. In blended learning classes, it is important to concentrate on assessing and evaluating student performance, paying attention to both academic performance and the development of students' learning abilities.

Setting up a scientific and reasonable evaluation system of blended teaching effect is predicated on accurately positioning the evaluation objects and goals. The main focus of this study's evaluation of the teaching effect is the students, who are also fully acknowledged for their central role in the learning process in the classroom [10]. It is important to consider both the effects of online and offline classroom learning when evaluating a teacher's teaching effectiveness in order to do so scientifically and accurately. The evaluation of the impact of blended learning takes into account various indicators, such as the level of student engagement in the online classroom, homework completion, and other factors [11].

### 2.2. Construction of the Indicator System

#### 2.2.1. Initial Establishment of the Evaluation Index System of Blended Teaching Effect

When constructing the system, in order to achieve a more accurate and scientific evaluation effect, sufficiently clear indicators and no duplication should be selected [12]. In the system structure of this study, the selected index systems mainly include learning attitude, learning performance, academic ability, and practical innovation ability. These four index systems are used as the first-level indicators, and at the same time, the first-level index system is further divided into several more specific indicators. These indicator systems are all secondary indicators, the specific structure is given in Figure 1.

#### 2.2.2. Screening Evaluation Indicators

In this study, the Delphi method was used to filter the evaluation indicators.

The filtering steps are as follows:

1. Setting up a coordination group to assign tasks to each person;
2. Determining the object of inquiry. Usually, well-known experts with rich experience were chosen;
3. Drawing up a consultation form and recording the relevant content and background information to be consulted.
4. Recording and analyzing the opinions of the first round of experts;
5. Second round of consultation with experts;
6. By comparing the results of the two rounds of expert consultation and making a reasonable analysis, comprehensively select the evaluation indicators for the quality of blended teaching.

#### 2.2.3. Calculation Method of Relevant Indicators

*(1) Expert Authority Level S_*t*_*. The authority of experts is very important to the reliability of the assessment, so it is necessary to consider the authority of the corresponding experts for a certain indicator, so as to process the evaluation results more accurately [13]. The degree of authority of an expert is usually determined by two factors: one is the expert's proficiency *S*_*a*_ on a certain issue, and the other is the basis of the expert's judgment *S*_*b*_. The formula for calculating the authority of an expert is shown in formula:

(1) $$\begin{array}{c} S_{t}=\frac{S_{a}+S_{b}}{2}. \end{array}$$

*(2) Weighted Arithmetic Mean S_*n*_*. The higher the weight of the index element, the greater the importance, then the weighted average arithmetic value is larger. Its main significance is to reflect the concentration of experts' scores and its formula is shown in formula:

(2) $$\begin{array}{c} S_{n}=\frac{1}{i}\sum_{m=1}^{i}S_{t}S_{nm}. \end{array}$$

In the formula: *S*_*n*_—the arithmetic weighted average of element *n*; *S*_*nm*_—the rating value of the expert *m* to the element *n*; *i*—the number of experts.

*(3) Full Score Frequency Q*. The frequency of full score refers to the comparison between the number of experts *i*_n_ who give full marks to each index element and the total number of experts *i* who make evaluations. The formula is as follows:

(3) $$\begin{array}{c} Q=\frac{i_{n}}{i}. \end{array}$$

*(4) Grade and T_*n*_*.

(4) $$\begin{array}{c} T_{n}=\sum_{n=1}^{S_{n}}S_{nm}. \end{array}$$

In the formula: *S*_*nm*_—the evaluation level of the index element *m* by expert *n*.

*(5) Coefficient of Variation V_*n*_*. Another key indicator for evaluating the degree of volatility is the coefficient of variability, which represents the different degrees of cognition of the importance of the index element *n* by different experts. That is to say, the smaller the coefficient of variability, the smaller the difference in cognition among experts, and the more coordinated the evaluation process.

*(6) Expert Opinion Coordination Coefficient R*. The larger the opinion coordination coefficient, the smaller the evaluation difference among all experts, and the higher the coordination degree between experts. The value range of the coefficient is between 0 and 1. The calculation formula is shown in formula (5):

(5) $$\begin{array}{c} R=\frac{12}{i^{2}\left(j^{3}-i\right)-i\sum_{n=1}^{i}t_{n}}\sum_{n=1}^{i}e_{n}^{2}, \end{array}$$

(6) $$\begin{array}{c} \sum_{n=1}^{i}e_{n}^{2}=\sum_{n=1}^{i}{\left(P_{n}-\bar{P}\right)}^{2}. \end{array}$$

In these formulas: *e*_*n*_^2^—the deviation of the evaluation level of the expert to the index element *n*; *i*—the total number of indicator elements; *P*_*n*_—the evaluation level sum of index element *n*; $\bar{P}$—the mean value of the sum of the evaluation grades of all the index elements.

(7) $$\begin{array}{c} d_{i}=\sum_{l=1}^{L}\left(d_{l}^{3}-d_{l}\right). \end{array}$$

In the formula, *L*—the same number of groups in the expert evaluation value;*d*_l_—the same number of ranks in the group.

Significance test of coordination coefficient:

(8) $$\begin{array}{c} x^{2}=\frac{1}{ij\left(j+1\right)-1/j-1\sum_{n=1}^{i}D_{n}}\sum_{n=1}^{j}e_{n}^{2}. \end{array}$$

*(7) Expected Value of Indicators*. The expected value needs to be obtained through the rank, weighted average, coefficient of variation, and full score frequency of each index element according to the “equal probability principle,” so as to evaluate the importance of each index element [14].

### 2.3. Determination of the Weight of the Evaluation Index of the Blended Teaching Effect

#### 2.3.1. Analytic Hierarchy Process

*(1) Theoretical Concepts*. AHP is an analytical method that combines qualitative and quantitative analysis, systematization, and hierarchy [15]. It can quantify and model decisions in complex systems. Decision-makers need to decompose complex problems into multiple factors and multiple levels, and then select the optimal solution based on the weights of these factors [16]. This method is very effective and real-time in dealing with complex problems, and has been widely used all over the world. The flow chart of AHP is shown in Figure 2.

*(2) Determination of the Weights of Indicators at All Levels*. Determination of the weight of the first-level indicator:

At the same level, experts judge the importance of two different index elements. Then they judge the value of the scale, which is taken according to the score scale, and finally, the corresponding judgment matrix can be generated [17]. After the decision matrix generating, the relevant importance is calculated. The sum-product method is used in this study, and the calculation process is as follows:

Matrix *B* is column normalized:

(9) $$\begin{array}{c} a_{nm}=\frac{b_{nm}}{\sum_{n=1}^{i}b_{nm}}\left(n,m=1,2,3\ldots i\right). \end{array}$$

The rows are added to get ${\bar{R}}_{n}$:

(10) $$\begin{array}{c} {\bar{R}}_{n}=\sum_{n=1}^{i}a_{nm}. \end{array}$$

Normalizing the rows gives the weight coefficient *R*_*n*_:

(11) $$\begin{array}{c} R_{n}=\frac{{\bar{R}}_{n}}{\sum_{n=1}^{i}{\bar{R}}_{n}}. \end{array}$$

The consistency of the matrix is judged and tested. Assuming that *α*max is the maximum eigenvalue of the judgment matrix *B*, and the judgment calculation formula of the maximum eigenroot is:

(12) $$\begin{array}{c} \alpha_{\max}=\frac{1}{i}\sum_{n}\frac{{\left(\text{BR}\right)}_{n}}{R_{n}},\\ \text{CI}=\frac{\alpha_{\max}-i}{i-1}. \end{array}$$

When *i* = 4, the consistent average random index RI can be obtained through the index parameters given in Table 1, and the consistency ratio can be calculated according to the obtained value:

(13) $$\begin{array}{c} \text{CR}=\frac{\text{CI}}{\text{RI}}. \end{array}$$

The consistency of the matrix is unsatisfactory in the case of CR > 0.1, demonstrating the unreliability of the first-level indicators' weight. On the other hand, the model's outcomes are consistent, meaning that the weights assigned to the first-level indicators are reliable and effective. The weight value of each first-level indicator can then be calculated.

Determination of secondary indicator weights:

According to the steps of the first-level indicators mentioned above, the AHP is also used to check the consistency of the teacher's teaching effect evaluation index system and calculate the weights of the second-level indicators [18].

#### 2.3.2. Calculation of Combined Weights

The formula for calculating the combined weight of the secondary indicators is:

(14) $$\begin{array}{c} R=R_{n}\Delta R_{nm}. \end{array}$$

In the formula: *R*_*nm*_—the weight of the secondary index; *R*_*n*_—the weight of the primary indicator to which the secondary indicator belongs.

All combined weights should add up to 1. Generally speaking, in the construction process of the judgment matrix, each expert's focus is different. Many judgment matrices will likely exist at the same time. Therefore, it can be solved by means of a weighted average, and the final weight of each level can be obtained.

### 2.4. Kirkpatrick Evaluation Model

#### 2.4.1. Introduction to the Model

The reaction layer, the learning layer, the behavior layer, and the result layer are the four layers that make up the Kirkpatrick model. Among these four levels, the response layer primarily assesses students' feedback on classroom instruction; the learning layer assessment assesses students' performance in the classroom; the behavior layer primarily looks at students' mastery of the knowledge they have learned; and the function of the outcome layer primarily assesses students' self-expression in the classroom [19].

As the model's four levels are evaluated, the evaluation difficulty will increase. Questionnaires, role-playing, and interview questions are just a few of the many evaluation techniques that can be used [8]. Activities for various levels of evaluation can be carried out by using these methods in their entirety. More focus should be placed on changes that occur before and after trainer training.

#### 2.4.2. Establishing a Blended Teaching Effect Evaluation System Based on the Kirkpatrick Model

In this study, the Kirkpatrick evaluation model was introduced and combined the characteristics of the current blended learning to construct a blended teaching effect evaluation framework [20].

*(1) Reaction Layer Evaluation*. The evaluation of the response layer is mainly about the feedback and satisfaction of the students with the teaching method. A very enthusiastic and highly motivated learning atmosphere can improve the learning effect of a certain project. The evaluation can be carried out from three dimensions: course teaching content and teaching form, teachers' evaluation, and teaching environment. These dimensions can also be subdivided. At the same time, different evaluation methods can be used to investigate the evaluation objects. The survey time can be selected at the end of the period.

*(2) Learning Layer Evaluation*. The main goal of this layer's evaluation is to gauge how well students learn when taught in offline classrooms and online classrooms, respectively. This link is crucial for assessing the effectiveness of blended learning because it can directly reflect how the mode of instruction affects learning. More observational indicators, such as the capacity for independent and cooperative learning, the mastery of professional knowledge and skills, and other factors, should be taken into account when evaluating the blended teaching model, which combines online and offline teaching.

*(3) Behavioral Layer Evaluation*. The assessment of the behavioral level is mainly aimed at students' proficient use of teaching content, that is, the behavioral changes of students caused by blended teaching. The focus of the evaluation is to evaluate the behavior of students in the mixed teaching model, thus making it a long time and dynamic evaluation process. It is necessary to conduct long-term observations of students' behavior changes. The main observation targets are students' attitude changes, behavior changes, and concept changes. When processing and analyzing the results, the differences in students' behavior before and after the change of learning mode should be focused on.

*(4) Results Layer Evaluation*. The evaluation at the result level primarily reflects the students' academic performance. Final tests and other methods of evaluation are frequently employed. The results of the students' academic accomplishments can be seen clearly in their test scores. Based on the students' entry scores and any certificates they received during a particular semester, it is also possible to perform a more in-depth analysis. Students can use their newly acquired knowledge and skills on other projects while participating effectively in this blended learning environment. This is a prolonged process. As a result, the end-level evaluation in the evaluation system proposed in this study should take place 6 months after the conclusion of the blended learning. It is important to consider the evaluation's timeliness in order to ensure a more thorough and accurate final assessment.

In order to make the blended teaching effect evaluation system based on the Kirkpatrick model easy to understand, the summary framework made in this study is shown in Table 2.

#### 2.4.3. Recommendations for the Use of the Kirkpatrick Evaluation Model

The relationship between the four evaluation levels of the Kirkpatrick evaluation model is progressive, as shown in Figure 3. It can be seen that the operation difficulty between the levels is increasing, the evaluation time is becoming longer, and the effect is becoming more and more obvious. Under the theoretical guidance of the Korotkoff evaluation model, when colleges and universities conduct blended teaching effect evaluation, they should start from the classroom as a whole. They should clarify the relationship between students' learning and the realization of teaching goals. It should be determined which stage and what level of evaluation need to be used. There are two ways to better use the Kirkpatrick model when evaluating the effect of blended teaching.

*(1) Select the Appropriate Tool*. Different survey methods should be correctly selected at different levels. For example, forums and surveys can be used for the reaction layer; competitions and written tests can be used for the evaluation of the learning layer; students' online self-evaluation and online teacher evaluation and other methods can be used for the evaluation of the behavioral layer; the evaluation at the result level can use self-evaluation questionnaires or final academic performance.

*(2) Pay Attention to the Evaluation Results*. In the process of using the Kirkpatrick evaluation model, pay attention to and communicate with the feedback information of the evaluation results received. Then analyzing the evaluation results, exploring the advantages and disadvantages of the teaching model then revising and improving the blended teaching model continuously. In this way, the Korotkoff evaluation model can be used more fully to achieve the purpose of improving the teaching effect.

## 3. Experiment Results of Blended Teaching

This study conducted an experimental investigation on the teaching effect of a university that conducted blended teaching. First, the commonly used analytic hierarchy process was used to evaluate the blended teaching effect of the university. In the selection of evaluation indicators, consultations were initiated with 15 authoritative experts in the field of teaching. In this way, expert opinions were collected, the results were sorted out, and the authority level of experts was obtained.

It can be clearly seen from Table 3 that the authority degree of experts in each of the four groups of first-level indicators was greater than 0.8. *S*_*t*_ > 0.8 indicated that the authority of the 15 authoritative experts consulted in the experimental investigation of this study was very high and the survey results were accurate and credible. In addition, a survey was conducted on the degree of coordination of opinions of experts, and the coordination coefficients and degrees of freedom of indicators at all levels were obtained. It is found that the coordination coefficients were all greater than 0.18. The data showed that the degree of coordination of opinions among 15 authoritative experts was very high, which made the experimental results more credible. The experimental data is as follows.

From the survey data, it can be seen from Table 4 that the 15 experts have a high degree of authority and coordination of opinions, and the opinions of the experts were relatively accurate. However, in order to compare the index differences between online and offline and blended teaching models, this study used AHP and the Kirkpatrick model to make experimental comparisons. The experimental data are as follows.

The data in Figure 4 is the comparison of the weights of the evaluation system indicators under the online, offline, and blended teaching modes calculated by the AHP. It can be seen that the learning ability has the largest weight in the evaluation indicators of the online teaching mode, and the weight value is 0.376. Among the evaluation indicators of the lower teaching mode, the learning ability is also the most weighted, with a weight value of 0.373. The largest weight in the evaluation indicators of the blended teaching mode is the practical ability, with a weight value of 0.46. Comparing the data, it can be seen that the teaching evaluation system of the online and offline teaching modes of the university pays attention to the learning ability of the students, while the hybrid teaching effect evaluation system pays more attention to the practical ability of the students, and the students' academic performance evaluation is a small part.

The data in Figure 5 showed the weights of the first-level indicators in the teaching effect evaluation system based on the Kirkpatrick evaluation model. The data showed that the behavior layer and the result layer have the largest weights in the evaluation indicators of the offline teaching mode. The weight values are 0.33 and 0.34 respectively; the largest weights in the online evaluation index are the learning layer and the behavior layer, and the weight values are 0.36 and 0.31, respectively. The largest weight in the hybrid mode evaluation index are the learning layer and the result layer, the weight value both are 0.3. In contrast, it can be seen that, for the teaching effect evaluation system based on the Kirkpatrick four-level evaluation model, the traditional offline teaching mode pays more attention to the students' practical ability and final academic performance in the classroom teaching evaluation. It regards these two points as important indicators of the effectiveness of classroom teaching. The recently emerging blended teaching currently pays more attention to the students' learning ability and learning results in the classroom. Whether the students' learning ability of the blended classroom teaching has improved, it can decide whether to continue the blended teaching mode.

In order to compare the impact of the two evaluation models on the evaluation of the effect of blended teaching, this study compared the evaluation systems of the mixed teaching effect under the two models. The experimental survey data are as follows:

From the experimental data in Figures 6 and 7, it can be seen that the weights of the final combined evaluation indicators in the hybrid teaching effect evaluation system under the two models were very close. Those with a large proportion of weights were concentrated on the evaluation of practical ability. The maximum weight was the innovation evaluation of course papers, and the weights of evaluation indicators were all greater than 0.15; The evaluation index of the teaching effect evaluation system based on AHP has the smallest weight of the number of platform logins, and the weight value is 0.022, while the Kirkpatrick evaluation model is 0.011.

Although the two blended teaching effect evaluation systems differ in numerical value, the overall evaluation indicators focus on roughly the same that they both focus on the evaluation of students' theoretical innovation and extracurricular practical ability.

For the blended teaching model, evaluating the effectiveness of classroom teaching focuses on the practical ability of the students. Only by transforming classroom knowledge into practical application can reflect the success of the teaching effect. Although the evaluation weight of learning attitude in blended learning is not high, it is also one of the indispensable evaluation indicators.

## 4. Conclusion

This study established a mixed teaching effect evaluation system on the basis of the Kirkpatrick evaluation model, conducting a preliminary exploration of the teaching effect evaluation of the mixed teaching model. It conducted an experimental investigation. In the experimental investigation, this study used both AHP and Kirkpatrick evaluation model-based teaching effect evaluation framework to compare the evaluation effect. Through the experimental comparison of the two evaluation systems, the following conclusions can be drawn:

1. Compared with the evaluation system based on AHP with an expert authority greater than 0.8, the blended teaching effect evaluation system based on the Kirkpatrick evaluation model has a similar trend in the weights of evaluation indicators. It indicated that the blended teaching effect evaluation system based on the Kirkpatrick evaluation model also has scientific and accurate evaluation results, and has a high credibility of teaching effects.
2. Compared with the AHP model, the Kirkpatrick assessment model is more clear and simple. It can clearly show the relationship and focus of indicators at all levels of the effect of blended teaching.

However, it is not difficult to see from the experimental investigation of this study that there are still some problems in the experiment. For example, it does not take into account the subjectivity and independence of the mutual evaluation between teachers and peers, which makes the evaluation results lack credibility. And students' poor judgment ability is easy to be influenced by the surroundings and other problems such as follow-up evaluation and so on. Therefore, in response to these problems, the blended teaching effect evaluation system still has research value and great significance in the future.

## Figures and Tables

**Figure 1:** Composition diagram of blended learning evaluation indicators.

**Figure 2:** AHP flow chart.

**Figure 3:** Kirkpatrick model teaching effect evaluation index system.

**Figure 4:** Weights of first-level indicators in different modes.

**Figure 5:** Weights of the first-level indicators of the kirkpatrick model.

**Figure 6:** Secondary indicator weights under the two models.

**Figure 7:** The final combination weight diagram of the blended teaching effect evaluation system.

**Table 1:** Average random consistency index.

Order	1	2	3	4	5	6	7	8	9
RI	0	0	0.58	0.9	1.12	1.24	1.32	1.41	1.45
CI	0	0	0.174	0.42	0.98	1.10	1.21	1.22	1.34

**Table 2:** Basic framework of blended teaching effect evaluation system based on Kirkpatrick model.

Evaluation level	Evaluation metrics	Evaluation method	Evaluation time
Reactive layer	Teachers, courses, environment	Satisfaction questionnaire personal interview	Before the end of blended teaching
Learning layer	Self-learning concept, professional knowledge, professional skill	Self-assessment exam in-depth interview	Blended teaching process
Behavioral layer	Behavioral changes, attitude change, concept change	Questionnaire survey in-depth interview	Three months after blended teaching
Result layer	Personal achievement	Questionnaire standardized test	Blended teaching ends between 6 months and 1 year

**Table 3:** Evaluation form of expert authority.

First-level indicator											
Learning attitude			Learning ability			Practical ability			Academic performance		
*S*_*a*_	*S*_*b*_	*S*_*t*_	*S*_*a*_	*S*_*b*_	*S*_*t*_	*S*_*a*_	*S*_*b*_	*S*_*t*_	*S*_*a*_	*S*_*b*_	*S*_*t*_
0.83	0.85	0.86	0.90	0.75	0.83	0.75	0.91	0.84	0.84	0.91	0.84

**Table 4:** Degree of coordination of expert opinions.

	Coordination coefficient	*C* ^2^	Degrees of freedom	Sig.
First-level indicator	0.187	16.403	4	0.002
Secondary indicators	0.195	104.658	11	0.000

## Data Availability

The data used to support the findings of this study are available from the corresponding author upon request.
